# Regulatory Effects of *Lycium barbarum* Extract and Isolated Scopoletin on Atopic Dermatitis-Like Skin Inflammation

**DOI:** 10.1155/2022/2475699

**Published:** 2022-09-15

**Authors:** Seon Gyeong Bak, Hyung-Jin Lim, Yeong-Seon Won, Soyoung Lee, Sun Hee Cheong, Seong Jin Lee, Eun Young Bae, Seung Woong Lee, Seung Jae Lee, Mun-Chual Rho

**Affiliations:** ^1^Functional Biomaterial Research Center, Korea Research Institute of Bioscience and Biotechnology (KRIBB), Jeongeup 56212, Republic of Korea; ^2^Department of Marine Bio Food Science, Chonnam National University, Yeosu 59626, Republic of Korea; ^3^CHA MEDITECH Co., Ltd., 199 Techno 2-ro, Daejeon 34025, Republic of Korea; ^4^Elohim Co., Ltd, R&D Center, 199 Techno 2-ro, Daejeon 34025, Republic of Korea

## Abstract

*Lycium barbarum* and scopoletin are widely used in oriental Eastern medicine and are often consumed as teas. In this study, proinflammatory cytokines expressed in human keratinocytes (HaCaT) were induced by skin diseases caused by 2,4-dinitrochlorobenzene (DNCB) and tumor necrosis factor alpha (TNF-*α*)/interferon gamma (IFN-*γ*). The inhibitory activity of *L. barbarum* EtOH extract (LBE) and scopoletin on proinflammatory cytokines and chemokines was investigated. In the DNCB-induced animal model, oral administration of LBE inhibited skin lesions and proinflammatory cytokines and chemokines and showed inhibitory effects *in vitro*. Additionally, as a result of examining the efficacy of scopoletin isolated from *L. barbarum*, scopoletin in HaCaT cells showed inhibitory effects on proinflammatory cytokines and chemokines. It shows promise in the treatment of chronic skin diseases.

## 1. Introduction

*Lycium barbarum* is the mature fruit of *L. barbarum* vine, a deciduous shrub belonging to the *Solanaceae* family [1]. It is a red fruit that looks a small pepper, is used medicinally in oriental medicine, and is also consumed in large amounts as a tea for the purpose of health promotion. *L. barbarum* has been reported to have many antioxidant and anti-inflammatory effects [2], including inhibition of PC3 cell proliferation *in vitro* [3] and prevention of UVB-induced skin damage [4]. In addition, a component of *L. barbarum* attenuated type II collagen-induced arthritis [5]. Scopoletin (7-hydroxy-6-methoxycoumarin) is a coumarin derivative and is contained in many medicinal plants, such as *L. barbarum*, *Erycibe obtusifolia*, *Aster tataricus*, and *Foeniculum vulgare* [6]. A previous report showed that scopoletin had anti-inflammatory effects in the human mast cell line HMC-1 [7], anti-obesity and fatty liver inhibitory effects [8], hypoglycemic and hypolipidemic effects [1], and synergistic antifungal effects [9].

The main function of the skin is protection and defense against external stimuli. Persistent external skin irritation by irritants and allergens triggers the progression of atopic dermatitis toward skin inflammation [10]. Skin inflammation is largely divided into two types: acute and chronic inflammation. Acute inflammation is the initial reaction by the body that initiates healing, and chronic inflammation can cause various problems [11]. 2,4-Dinitrochlorobenzene (DNCB, a hapten)-induced atopic dermatitis is acute inflammation involving dendritic cells and macrophage activation resulting in dermal damage and edema [12]. An acute inflammatory state directly affects the course of dermatitis treatment [13], and appropriate treatment is important. Therefore, the development of natural drugs with high efficacy and few side effects is important.

Due to the pharmacological profile of *L. barbarum* extract and isolated scopoletin and its reported immunoregulatory properties, we hypothesized that *L. barbarum* extract and isolated scopoletin might have a therapeutic effect on atopic dermatitis, such as skin inflammation. The purpose of this study was, therefore, to test the therapeutic activity of *L. barbarum* extracts and scopoletin against skin inflammation and to elucidate the underlying therapeutic mechanisms of action, as part of our ongoing search for immunomodulatory medicines extracted from medicinal plants or edible plants.

## 2. Materials and Methods

### 2.1. Preparation of *L. barbarum* EtOH Extract (LBE) and Isolation of Scopoletin

*L. barbarum* (90 kg) was extracted with 30% (*v*/*v*) of EtOH in distilled water 720 L at 70°C (8 h). After filtering, the filtrate was concentrated under reduced pressure (60°C). The residue (65 Brix, 500 mL) was suspended in distilled water (3.5 L), and the aqueous layer was partitioned with EtOAc (3 L, 3 times). The EtOAc layer was concentrated under reduced pressure to obtain 2.06 g of extract. The EtOAc layer was subjected to MPLC column chromatography (column: C18 RediSepRf (130 g); flow rate 15 mL/min) eluted with MeOH (0-100%, *v*/*v*) to obtain 7 fractions (MP-1~MP-7). Fractions MP-3 (168.3 mg) and MP-4 (144.7 mg) were further purified by preparative HPLC (Phenomenex Luna C18 column 250 × 21.2 mm, 5 *μ*; flow rate 6 mL/min), using isocratic elution with CH_3_CN in H_2_O (18% CH_3_CN, 60 min) to scopoletin (5.4 mg). The structure of scopoletin was confirmed by 1H-NMR (500 MHz) and 13C-NMR (125 MHz) spectra obtained on a Bruker Biospin Avance 500 spectrometer (Bruker, Billerica, MA, USA) with CD3OD solvent.

*Scopoletin*, Amorphous solid; 1H NMR (500 MHz, CD3OD) *δ*H 7.84 (1H, d, J =9.5 10.0 Hz, H-4), 7.10 (1H, s, H-5), 6.76 (1H, s, H-8), 6.19 (1H, d, J =9.5 10.0 Hz, H-3), 3.90 (3H, s, OMe-6); 13C NMR (125 MHz, CD3OD) *δ*c 164.1 (C-2), 151.4 (C-7), 152.9 (C-9), 147.1 (C-6), 146.1 (C-4), 112.6 (C-3), 112.5 (C-10), 109.9 (C-5), 103.9 (C-8), 56.8 (OMe-6).

### 2.2. Animals

Female BALB/c mice (6 weeks) were purchased from Samtako (Osan, Korea). All animals had ad libitum access to standard rodent chow and filtered water during the study. The animals were housed (5 per cage) in a laminar air flow room maintained at a temperature of 22 ± 2°C and relative humidity of 55 ± 5%, with a 12 h light/dark cycle throughout the study. Care and treatment of the animals were conducted in accordance with the guidelines established by the Public Health Service Policy on the Humane Care and Use of Laboratory Animals and were approved by the Institutional Animal Care and Use Committee of the Korea Research Institute of Bioscience and Biotechnology.

### 2.3. Induction of DNCB-Induced Atopic Dermatitis-Like Lesions

A total of 25 mice were divided into five groups (*n* = 5): PBS topically applied to ear and PBS-treated group, DNCB applied and PBS-treated group, DNCB applied and LBE (100 or 300 mg/kg) treated groups, and DNCB applied and dexamethasone (DX, 5 mg/kg) treated group. During the first week of induction, DNCB (2%, 20 *μ*L/ear) was applied to each ear once for sensitization. Then, DNCB (1%, 20 *μ*L/ear, once) was challenged to both BALB/c mouse ears for 3 weeks. LBE (100 or 300 mg/kg) or DX (5 mg/kg) was orally administered by gavage for five consecutive days per week at the time of the DNCB challenge.

### 2.4. Histological Assay

Mouse ear tissues were fixed in 4% (*w*/*v*) paraformaldehyde in phosphate-buffered saline (PBS, pH 7.4). The fixed tissues were embedded in paraffin and cut into 4 *μ*m thick sections, which were stained with hematoxylin and eosin (H&E).

### 2.5. Cell Culture

The human keratinocyte cell line, HaCaT, was maintained in Dulbecco's Modified Eagle's Medium (DMEM), supplemented with 10% heat-inactivated fetal bovine serum (FBS) and 1% penicillin-streptomycin at 37°C, 90–95% humidity, and 5% CO_2_.

### 2.6. ELISA Analysis

Serum IgE, cytokine (TNF-*α*, IL-1*β*, IL-6, and IL-8), and chemokine (CCL17/TARC, CCL22/MDC) levels in the cell culture medium were determined using an enzyme-linked immunosorbent assay (ELISA) kit (Thermo Fisher Scientific, Waltham, Massachusetts, USA; BD Biosciences, San Diego, CA, USA; R&D Systems, Minneapolis, MN, respectively) according to the manufacturer's instructions. The absorbance was measured at 450 nm using a microplate reader.

### 2.7. Real-Time Quantitative PCR

Total RNA from HaCaT cells treated with LBE, scopoletin, cyclosporine A, and/or TNF-*α* (50 ng/mL)/INF-*γ* (50 ng/mL) or ear tissues of each group was isolated using TRIzol reagent. First-strand complementary DNA (cDNA) was synthesized using a PrimeScript 1st strand cDNA Synthesis Kit (Takara Bio Inc., Shiga, Japan). PCR was performed using a Bio-Rad T100 thermal cycler (Bio-Rad, Hercules, CA, USA) according to the manufacturer's protocol. In brief, real-time PCR was performed by a StepOnePlus Real-Time PCR System using TaqMan probes and TaqMan Real-Time PCR master mix (Applied Biosystems, Foster City, CA, USA). 18S rRNA was used as an endogenous control for normalization. The following TaqMan primers and probes were purchased from Applied Biosystems, Thermo Fisher Scientific: TNF-*α* (Hs01113624_g1 and Mm00443258_m1), interleukin- (IL-) 1*β* (Hs01555410_m1 and Mm00434228_m1), IL-6 (Hs00174131_m1 and Mm00446190_m1), IL-8 (Hs00174103_m1), CCL17 (Hs00171074_m1 and Mm01244826_g1), and CCL22 (Hs01574247_m1 and Mm00436439_m1).

### 2.8. Western Blot

Total protein was extracted as previously described [14]. HaCaT cells (1 × 10^6^ cells/well in 6-well plates) were pretreated with LBE, scopoletin, or cyclosporine for 1 h and then stimulated with TNF-*α* (50 ng/mL)/IFN-*γ* (50 ng/mL) for 30 min. The cells were lysed with 100 *μ*L of cell lysis buffer (Cell Signaling Technology, Danvers, MA, USA). The lysed samples were vortexed, incubated for 30 min on ice, and centrifuged at 13,000 rpm for 10 min at 4°C. The supernatants were collected and quantified using a DC protein assay kit (Bio-Rad, Contra Costa County, CA, USA). The nuclear protein of HaCaT cells was extracted as described previously [14]. Equal amounts of protein lysate were subjected to electrophoresis on an 8–12% SDS-PAGE gel, and the protein bands were then transferred to a polyvinylidene fluoride (PVDF) membrane. After blocking with 5% bovine serum albumin in Tris-buffered saline, the membrane was incubated with the target primary antibody, washed, and subsequently incubated with anti-IgG horseradish peroxidase-conjugated secondary antibody. The results were developed using a West-Queen RTS Western Blot Detection Kit (iNtRON Bio, Seongnam, Korea). The following antibodies were purchased from Cell Signaling Technology: p-p38 (#4511S, rabbit monoclonal, 1: 1000), p38 (#8690S, rabbit monoclonal, 1 : 1000), p-ERK (#9101S, rabbit monoclonal, 1 : 1000), ERK (#4348S, rabbit monoclonal, 1 : 1000), actin (#4967S, rabbit monoclonal, 1 : 1000), and phospho-NF-*κ*B (#3033S, rabbit polyclonal, 1 : 1000); the following were purchased from Santa Cruz: p-JNK (#sc-6254, mouse polyclonal, 1 : 1000), JNK (#sc-7345, mouse polyclonal, 1 : 1000), p-Stat1 (#sc-8394, mouse polyclonal, 1 : 1000), and Lamin B (#sc-6216 goat polyclonal, 1 : 1000).

### 2.9. Statistical Analysis

Statistical analysis was performed using Prism 5 software (GraphPad Software, San Diego, CA, USA). The data are presented as the mean ± SD of nine individual experiments. Statistical significance was determined by one-way ANOVA followed by Tukey's test for multiple comparisons.

## 3. Results

### 3.1. Effect of LBE in DNCB-Induced Atopic Dermatitis

To evaluate the antiatopic effects of LBE, a DNCB-induced atopic dermatitis animal model was used. DNCB is a powerful material for the induction of atopic lesions [12]. As shown in Figure 1(a), atopic skin lesions in the DNCB-treated group were significantly aggravated. The histopathological pathology analysis using H&E staining showed an increase in edema and immune cell infiltration. In addition, ear thickness was increased with DNCB treatment (Figure 1(b)). However, oral administration of LBE decreased the DNCB-induced atopic skin lesions (Figures 1(a) and 1(b)). IgE is an immunoglobulin associated with Th2 responses in atopic dermatitis [12]. The DNCB-treated group showed significantly increased serum IgE levels. However, oral administration of LBE decreased serum IgE levels (Figure 1(c)). In atopic dermatitis, damaged epithelial cells and keratinocytes produce proinflammatory cytokines and chemokines such as TNF-*α*, IL-1*β*, IL-6, IL-8, CCL17, and CCL22 [15]. To assess the anti-inflammatory effect of LBE on atopic dermatitis, the gene expression of proinflammatory cytokines and chemokines was determined in ear tissues. The DNCB-treated group showed markedly elevated proinflammatory cytokine and chemokine levels, such as IL-1*β*, IL-6, IL-8, CCL17, and CCL22. However, oral administration of LBE alleviated gene expression levels (Figure 2). Our data indicated that LBE attenuates Th2-mediated atopic dermatitis-related skin lesions.

### 3.2. Effect of LBE on Proinflammatory Gene Expression in HaCaT Cells

To determine the anti-inflammatory effect of LBE at the cellular level, proinflammatory cytokine and chemokine expressions under TNF-*α*/IFN-*γ*-induced inflammation in HaCaT human keratinocytes were analyzed. HaCaT cells were pretreated with various concentrations of LBE (10, 30, and 60 *μ*g/mL) for 1 h before stimulation with 50 ng/mL TNF-*α*/IFN-*γ* treatment. TNF-*α*/IFN-*γ*-stimulated HaCaT cells showed high levels of proinflammatory factors, TNF-*α*, IL-1*β*, IL-6, IL-8, CCL17 and CCL22 gene expression and production. However, pretreatment with LBE inhibited TNF-*α*/IFN-*γ*-stimulated proinflammatory gene expression and production in a concentration-dependent manner (Figures 3 and 4). Our data showed that LBE inhibited inflammatory gene expression in keratinocytes.

### 3.3. Effect of LBE on Intracellular Signaling in HaCaT Cells

To demonstrate the mechanism of LBE on anti-inflammatory efficacy, the TNF-*α*/IFN-*γ*-stimulated intracellular signaling pathway was evaluated. MAPKs, including p38, EKR, and JNK, have shown a wide spectrum of bioactivities, such as cell cycle, metabolism, and inflammation activities at the cellular level [16]. STAT1 drives to Th2 responses, leading to the development of atopic dermatitis [17]. NF-*κ*B is a major transcription factor and plays critical roles in inflammatory gene expression [18]. Therefore, MAPKs, STAT1, and NF-*κ*B are treatment targets for inflammatory responses. TNF-*α*/IFN-*γ*-stimulated HaCaT cells showed elevated phosphorylation of signaling molecules such as p38, ERK, JNK, STAT1, and NF-*κ*B. However, pretreatment with LBE suppressed the TNF-*α*/IFN-*γ*-stimulated phosphorylation of signaling molecules (Figure 5). *β*-Actin and Lamin B were used as loading controls in the whole and nuclear proteins, respectively. Our data indicated that LBE downregulated the inflammatory-associated signaling molecules, leading to anti-inflammatory efficacy.

### 3.4. Effect of Scopoletin on Proinflammatory Gene Expression in HaCaT Cells

To verify the mode of action of LBE, we purified the LBE into fractions and single compounds. Scopoletin is an abundant molecule in natural products such as *Lycium barbarum* and has been reported various pharmaceutical activities [3, 9, 19–21]. The HaCaT cells were pretreated with various concentrations of scopoletin (5, 10, and 50 *μ*M) for 1 h before the stimulation. TNF-*α*/IFN-*γ*-stimulated HaCaT cells showed the increase of proinflammatory gene expression and production such as proinflammatory cytokines and chemokines. However, pretreatment of scopoletin suppressed the TNF-*α*/IFN-*γ*-stimulated proinflammatory gene expression and productions in a concentration-dependent manner (Figures 6 and 7). Moreover, the highest concentration of scopoletin showed an inhibitory efficacy similar to that of the positive control drug, cyclosporine A. Our data showed that scopoletin strongly regulated inflammatory gene expression in keratinocytes.

### 3.5. Effect of Scopoletin on Intracellular Signaling in HaCaT Cells

To inspect the mechanism of action of scopoletin, the TNF-*α*/IFN-*γ*-stimulated intracellular signaling pathway was evaluated. TNF-*α*/IFN-*γ*-stimulated HaCaT cells showed an increase in the phosphorylation of signaling molecules. However, pretreatment with scopoletin suppressed the TNF-*α*/IFN-*γ*-stimulated phosphorylation of signaling molecules (Figure 8). Furthermore, the highest concentration of scopoletin significantly suppressed the phosphorylation of MAPKs, STAT1, and NF-*κ*B. Our data indicated that scopoletin strongly regulates atopic skin lesions by controlling the inflammatory responses of keratinocytes.

## 4. Discussion

In this study, we investigated the inhibitory effects of *L. barbarum* and scopoletin on chronic inflammatory skin conditions. First, the anti-inflammatory activity of LBE was confirmed using an animal model of DNCB-induced dermatitis. LBE reduced DNCB-induced atopic like-skin lesions, such as increases in epidermal thickness and serum IgE levels. Additionally, LBE treatment inhibited the DNCB-induced gene expression of proinflammatory cytokines and chemokines. In HaCaT cells, TNF-*α*/IFN-*γ*-stimulated mRNA expression and protein secretion were verified for the anti-inflammatory activity of LBE on proinflammatory cytokine and chemokine levels, and the activity of scopoletin isolated from LBE showed similar activity. Moreover, the anti-inflammatory effects of LBE and scopoletin were demonstrated through the regulation of intracellular signaling pathways, including MAPKs, STAT1, and NF-*κ*B.

Atopic dermatitis is a complicated skin barrier disease characterized by immune hypersensitivity reactions caused by infiltration and activation of immune cells (lymphocytes, eosinophils, mast cells, etc.), resulting in skin lesions (dry skin, itchiness, eczema, erythema, etc.), dermal damage, keratinocytes inflammation, and skin remodeling [22]. To evaluate the treatment effect of LBE on atopic dermatitis-like skin inflammation, we used a DNCB-induced skin inflammation mouse model. The activation of dendritic cells and macrophages in the subcutaneous layer occurs after DNCB exposure, causing damage and inflammation of the skin layer through the secretion of proinflammatory cytokines and chemokines [23, 24]. Many previous studies consider that inflammatory responses are a target of therapeutic targets and that drugs from natural products should be developed [23, 25]. Therefore, verification of the efficacy of natural compounds for atopic dermatitis using the DNCB atopic model is appropriate for discovering new therapeutic substances. In this study, it was confirmed that after administration of LBE, changes in skin inflammatory properties were observed. Our data showed that oral administration of LBE, for 3 weeks, decreased the increase in epidermal thickness and the level of serum IgE in the DNCB-induced atopic dermatitis model. The gene expression of proinflammatory cytokines and chemokines was also suppressed by oral administration of LBE at the site of ear skin lesions.

Inflammatory stimuli such as TNF-*α*/IFN-*γ* are used in many skin disease studies because they can mimic the symptoms of atopic dermatitis such as skin inflammation in HaCaT cells [25]. In this study, LBE and scopoletin did not show toxicity on HaCaT cells in the experimental concentration range. LBE and scopoletin significantly inhibited the increase in the protein and mRNA levels of proinflammatory cytokines and chemokines in HaCaT cells stimulated with TNF-*α*/IFN-*γ*. Scopoletin has been reported to have an anti-inflammatory effect in HMC-1 cells [7], and the efficacy on mast cell-mediated allergic inflammation may be speculated. To understand the immune regulatory mechanisms, we investigated the effects of LBE and scopoletin on the MAPKs, STAT-1, and NF-*κ*B signaling pathways. Our results suggest that the anti-inflammatory and protective effects of LBE and scopoletin were due to inhibition of the production of proinflammatory cytokines and chemokines through suppression of the MAPKs, STAT1, and NF-*κ*B signaling pathways.

In conclusion, LBE ameliorated atopic dermatitis-like skin lesions in a DNCB-treated mouse model and inhibited proinflammatory cytokines and chemokines *in vivo* and *in vitro*. In addition, LBE induces anti-inflammatory effects by upregulating MAPKs, STAT1, and NF-*κ*B signaling in HaCaT cells stimulated with TNF-*α*/IFN-*γ*. Scopoletin isolated from LBE also downregulates inflammatory cytokines and chemokines in TNF-*α*/IFN-*γ* stimulated HaCaT cells and induces anti-inflammatory effects by regulating MAPKs, STAT-1, and NF-*κ*B signaling. Taken together, *L. barbarum* and scopoletin for the treatment of chronic skin inflammation represent new possibilities for natural drug development.

## Figures and Tables

**Figure 1:** Effect of LBE on skin lesions and IgE levels in DNCB-induced atopic dermatitis mouse model. (a) Skin lesions of the ear in DNCB-induced atopic dermatitis mice. Mice were sensitized by topically applied to both ears with 20 *μ*L of 2% DNCB. After a week, the mice were topically applied to both ears with 20 *μ*L of 1% DNCB for 5 times for a week for 3 weeks. LBE (100 or 300 mg/kg) or DX (5 mg/kg) was orally administered by gavage for five consecutive days per week at the time of 1% DNCB treatment. The image shows ear skin 24 h after the last treatment of DNCB. (b) Ear thickness with DNCB-treated was measured at the time of the 24 h after last of DNCB treatment using a digital ear thickness gauge. (c) Serum IgE levels were measured by ELISA. Serum was collected immediately after sacrifice of DNCB-induced atopic dermatitis mice. ^∗^*p* < 0.05 compared with DNCB-induced group.

**Figure 2:** Effect of LBE on proinflammatory gene expression levels in a DNCB-induced atopic dermatitis mouse model. Total RNA was extracted from ear tissues. The levels of proinflammatory cytokines such as IL-1*β*, IL-6, and IL-8 and chemokines such as CCL17 and CCL22 were measured by real-time quantitative PCR. ^∗^*p* < 0.05 compared with DNCB-induced group.

**Figure 3:** Effect of LBE on proinflammatory gene expression levels in TNF-*α*/IFN-*γ*-stimulated HaCaT cells. HaCaT cells were pretreated with 10, 30, and 60 *μ*g/mL LBE for 1 h before stimulation. Cyclosporin A, an immune suppressor, was used as a positive control drug. Then, HaCaT cells were stimulated with TNF-*α*/IFN-*γ* for 6 h, and RNA was extracted from the cells using TRIzol reagent. The levels of proinflammatory cytokines and chemokines were measured by real-time quantitative PCR. ^∗^*p* < 0.05 compared with TNF-*α*/IFN-*γ*-stimulated group.

**Figure 4:** Effect of LBE on proinflammatory cytokine secretion in TNF-*α*/IFN-*γ*-stimulated HaCaT cells. HaCaT cells were pretreated with 10, 30, and 60 *μ*g/mL LBE for 1 h before the stimulation. Then, HaCaT cells were stimulated with TNF-*α*/IFN-*γ* for 24 h and the supernatant was collected. The levels of secreted proinflammatory cytokines and chemokines were measured by ELISA. ^∗^*p* < 0.05 compared with TNF-*α*/IFN-*γ*-stimulated group.

**Figure 5:** Effect of LBE on intracellular signal transduction in TNF-*α*/IFN-*γ*-stimulated HaCaT cells. HaCaT cells were pretreated with 10, 30, and 60 *μ*g/mL LBE for 1 h before the stimulation. Then, HaCaT cells were stimulated with TNF-*α*/IFN-*γ* for 30 min, and whole proteins were extracted using Cell Signaling Technology total protein extraction reagent.

**Figure 6:** Effect of scopoletin on proinflammatory gene expression levels in TNF-*α*/IFN-*γ*-stimulated HaCaT cells. HaCaT cells were pretreated with 5, 10, and 50 *μ*M scopoletin for 1 h before the stimulation. Then, HaCaT cells were stimulated with TNF-*α*/IFN-*γ* for various time points, and RNA was extracted from the cells using TRIzol reagent. The levels of proinflammatory cytokines and chemokines were measured by real-time quantitative PCR. ^∗^*p* < 0.05 compared with TNF-*α*/IFN-*γ*-stimulated group.

**Figure 7:** Effect of scopoletin on proinflammatory cytokine secretion in TNF-*α*/IFN-*γ*-stimulated HaCaT cells. HaCaT cells were pretreated with 5, 10, and 50 *μ*M scopoletin for 1 h before the stimulation. Then, HaCaT cells were stimulated with TNF-*α*/IFN-*γ* for 24 h, and the supernatant was collected. The levels of secreted proinflammatory cytokines and chemokines were measured by ELISA. ^∗^*p* < 0.05 compared with TNF-*α*/IFN-*γ*-stimulated group.

**Figure 8:** Effect of scopoletin on intracellular signal transductions in TNF-*α*/IFN-*γ*-stimulated HaCaT cells. HaCaT cells were pretreated with 5, 10, and 50 *μ*M scopoletin for 1 h before the stimulation. Then, HaCaT cells were stimulated with TNF-*α*/IFN-*γ* for 30 min, and whole proteins were extracted using Cell Signaling Technology total protein extraction reagent.
